# Extraction of Intangible Cultural Heritage Visual Elements by Deep Learning and Its Application in Grassland Tourism of the Silk Road Culture

**DOI:** 10.1155/2022/3242960

**Published:** 2022-06-20

**Authors:** Xiangwei Bu, Mingyang Jiang

**Affiliations:** ^1^Academy of Fine Arts, Inner Mongolia Minzu University, Tongliao 028000, China; ^2^College of Computer Science and Technology, Inner Mongolia Minzu University, Tongliao 028000, China

## Abstract

Inner Mongolia is rich in grassland tourism resources, and the development of grassland tourism is of great significance to Inner Mongolia tourism and promotion of grassland protection. To better promote the grassland tourism of the Silk Road culture, the Conditional Global Area Network (CGAN) and Morphology Connected Component Chan-Vase (MCC-CV) algorithm are used to enhance and segment the traditional embroidery patterns in Inner Mongolia. Firstly, the generative adversarial network (GAN) is optimized, and a new GAN is proposed with the feature vector extracted from the convolutional neural network (CNN) as the constraint condition. Secondly, the automatic segmentation algorithm of embroidery based on the MCC-CV model is proposed, and finally, the proposed algorithm is tested. The test results demonstrate that after 8000 iterations of the proposed image-enhancement algorithm, its personalized features are enhanced, and the segmentation accuracy of the proposed image segmentation algorithm is 60%. The proposed algorithm provides some ideas for the application of deep learning (DL) technology in the grassland tourism of the Silk Road culture and also helps operators to accurately grasp the market and make tourists more comfortable and pleasant.

## 1. Introduction

Inner Mongolia is the main birthplace and carrier of grassland civilization. The vast Mongolian plateau has been a big stage for the activities of nomads in northern China since ancient times. The special region, special natural environment and production and lifestyle have created a unique grassland civilization. In the long-term production and life practice, the ancestors of the grasslands in the past dynasties not only left a large amount of material cultural heritage but also left a very rich and valuable intangible cultural heritage. However, with the development of the economy and the accelerated pace of modernization, intangible cultural heritage has been impacted by various cultural contents, and the environment in which it exists has also begun to deteriorate. This situation has attracted the attention of government departments, experts, and scholars [1, 2]. The development of grassland ecotourism can not only provide necessary material support for the protection of Mongolian intangible cultural heritage, but also provide a realistic need for the existence of intangible cultural heritage. Correctly handling the relationship between the development of grassland tourism and strengthening the protection of the intangible cultural heritage of ethnic minorities is very significant to achieve a win-win situation between the development of grassland ecotourism and the protection of Mongolian intangible cultural heritage [3, 4].

China is a multiethnic country, and each ethnic group has its own iconic elements. Scholars' creation and design of ethnic elements make ethnic-style works flourish in China. This not only promotes the combination of ethnic elements and artistic design but also opens up new paths for scholars to study. On the one hand, ethnic elements and modern art creation are closely related, and effective communication between the two can promote the development of national culture. On the other hand, national culture is also an important part of human culture and life, and the research on the collection, processing, and application of ethnic elements has also become a hot spot in the computer field. In contemporary society, handmade products with ethnic style such as embroidery are favored by many consumers. As a kind of national characteristic culture, embroidery art represents the style and the characteristics of the main ethnic elements in many regions. Embroidery art has been passed down from generation to generation, and some treasures are inevitably lost. Considering the cost-effectiveness of digital protection, the digital protection and exploration of embroidery culture should be included in the digital inheritance of national culture [5–7]. The grassland culture is formed and developed by the nomadic people in northern China in the process of facing the challenges from the natural environment or living environment of the grassland. It has six characteristics, namely, natural cultural nature; successive cultural trajectory; fluid cultural behavior; martial cultural psychology; open cultural essence; and honesty. It maintains the survival of the nomadic peoples, showing the vitality of nomads, and is an integral part of Chinese culture. Many researchers use deep learning (DL) techniques to study all the aspects of grassland culture, such as convolutional neural network (CNN) algorithms.

The innovation can be divided into two points. First, it proposes the generative adversarial network (GAN) data augmentation model based on embroidery image features as constraint rules. The model uses CNN to extract the basic texture features of the image and input them into the GAN. The network structure is optimized so that the generator can generate images with the texture features of the embroidery elements under the influence of the constraint rules. The improved model efficiency is significantly improved. Second, it proposes an automatic image segmentation method by fusing the Morphology Connected Component Chan-Vase (MCC-CV) model. The contribution is that most of the current artistic creations are created by using a large number of ethnic elements, with low practical value and very few creations close to life. The proposed network enables more applications for data augmentation and style transfer problems.

Section 1 provides an overview of the grassland tourism of the Silk Road culture and the protection of the intangible cultural heritage of ethnic minorities.  Section 2 discusses the research results, advantages, and disadvantages of the other researchers in this field.  Section 3 proposes an improved augmentation model of GAN data, and an automatic pattern segmentation method.  Section 4 designs the system and discusses the experimental environment and the data set used in the experiment.  Section 5 analyzes the experimental results, and Section 6 summarizes the whole work.

## 2. Literature Review

Researchers have also carried out a lot of research work in the related fields. Liu et al. [8] pointed out that fabric defect identification is an important means of quality control in textile mills, which uses deep convolutional neural networks (DCNN) to identify fabric defects with complex textures. To optimize DCNN, a new method is proposed to reveal the input patterns that initially induce specific activations in the network feature map, and the computational effort and a total number of parameters of the new network are 23% and 8.9% of the original model, respectively. Aiming at the problems of low accuracy and low efficiency of surface defect recognition of common woven fabrics, Liu et al. [9] proposed a fabric defect classification method based on unsupervised segmentation and extreme learning machine (ELM). The experimental results show that the proposed method has high classification accuracy and efficiency for fabric defect images and can better meet the requirements of practical applications. The work of Kumar and Bai [10] focuses on fabric analysis of complex designs, using color-based feature extraction to obtain global and local features, which are used as the input for fine-grained analysis of fabrics to perform fine-grained segmentation of the image. Jeyaraj and Samuel Nadar [11] developed a computer-aided fabric defect detection and classification method based on an advanced learning algorithm to classify fabric defects quickly and effectively. In the test task, the algorithm obtained an average accuracy of 94.85% and successfully identified 6 defects. Ji et al. [12] thought that traditional retrieval methods cannot achieve fast and accurate retrieval of fabric images. Therefore, a fabric image retrieval method based on multi-feature fusion was proposed, which can accurately analyze the characteristics of fabric images. Experiments indicate that using this method to retrieve fabric images can achieve better results. Yasar et al. [13] pointed out that defects during or after the weaving of the fabric can reduce the quality of the fabric, and proposed solutions to implement and automate the process under computer control. The authors segment the fabric image into equal-sized blocks to judge whether the fabric has defects. The fabric image is segmented into equal-sized blocks to judge whether the fabric is defective or not.

Giray et al. [14] investigated the perceptions of tourists in a small village called Kuyucak in southwestern Turkey, where rural tourism based on lavender production has recently developed. Results of an analysis of 175 questionnaires completed by online visitors showed that more than half of the respondents learned about the village through social media. Although the main purpose of their visit is nature/country experience and recreation/vacation, the main motivation for most is to take and share the photos through social media tools, which is a very important determinant of tourists' decisions and expectations. The results of the factor analysis indicated that the two components consisting of two variables, pre-visit perception and the physical condition of the village, together explained 65% of the overall satisfaction. The most vital component in a visitor's decision-making is their perception before the visit, meaning what they expect to see is more important than what they actually see, which represents visitor satisfaction. Allowing tourists to experience how they felt before visiting would contribute to the sustainability of the rural tourism activities, benefiting the region. Li and Wang [15] pointed out that the rapid development of industrial integration is conducive in optimizing the industrial structure. The integration of agriculture and tourism can promote the development of the agricultural economy and tourism economy. Based on the theory of industrial convergence, the necessity of the convergence of leisure agriculture and rural tourism is expounded. Finally, the development countermeasures are put forward: (1) more support from the government in policy, finance, and rural utilization is needed; (2) strengthen rural planning; (3) integrate agricultural resources; (4) establish incentive mechanism to attract talents. Liu [16] used an adaptive neural network algorithm to diagnose the industrial integration of rural cultural industry and rural tourism industry from the perspective of blockchain, taking cultural industry and rural tourism industry as examples. This will further consolidate the theoretical foundation for the integrated development of the tourism industry and the cultural industry and help promote the integrated development of the industry.

Nowadays, there are a lot of valuable literature results on the problem of automatic detection of fabric defects. However, the mature cloth inspection systems in foreign countries are used to detect defects in various yarns, natural fabrics, and other fabrics. These systems are expensive and still have missed detections and false detections. And these systems are not used in the research on the protection of the intangible cultural heritage of ethnic minorities. In addition, there are few researchers on grassland tourism, and researchers generally focus on rural tourism.

At present, the development of ethnic embroidery data has attracted the attention of people from all walks of life, but the data stored in the private sector is limited, and the dissemination is limited by regions and the development is slow. For the protection and inheritance of tie-dye culture, a low-cost and strong sharing method should be selected. The existing digital protection methods can record the tie-dye culture in detail through images, videos, etc., but if a large-scale project or work is carried out, the original data will face the problem of small-scale and insufficient training. Combining the current DL technology and image processing technology can effectively expand the data set of tie-dye images, which is of great help to the research and experimental training of experts and scholars.

## 3. Data-Enhanced Segmentation Technology of Grassland Silk Road Culture and Ethnic Embroidery Images

### 3.1. Research on Grassland Silk Road Culture

Mongolian embroidery techniques are unique, and there are four main types of typical techniques, namely embroidery, applique embroidery, plain embroidery, and engraving embroidery. Embroidery techniques mainly use colored silk threads, gold and silver threads, and various real silk threads as the main materials and embroider various patterns on the fabric one by one. Mongolian women do not need to use embroidery frames to embroider, but operate directly with both hands. There are three types of stitches most commonly used in embroidery, namely, plain stitches, contact stitches, and split stitches. This kind of stitching method can carefully paint the shape of flowers and birds, and the embroidered patterns are closer to nature, with simple composition and bright colors. A representative Mongolian embroidery pattern is shown in Figure 1.

The collection and digital protection of ethnic embroidery images have their own regional and ethnic limitations, and the amount of data stored is small and the scale is also small. The use of modern technology to realize the protection of tie-dye culture requires professional personnel to spend a lot of manpower and materials to collect and organize. If scholars want to combine national culture with DL projects, it will take a considerable amount of time for scholars and experts to find sufficient data. Choosing to use the method of GAN for unsupervised data augmentation training solves the problem of manpower and material resources to a certain extent. The generator model in the GAN has a relatively complex calculation process for other generative models such as Naive Bayes and mixture Gaussian models. The discriminator in the GAN is a simpler and more flexible structure with a single function [17]. In recent years, the development prospects of discriminative models are also very good, and they are widely used in recognition and detection. The GAN is an unsupervised learning process, the discriminator optimizes itself and approximates the distribution during the detection process, and does not need to be pre-defined. Lv et al. proposed an automatic online assessment method for cyber-physical system (CPS) reliability.

### 3.2. Data-Enhanced Segmentation Technology of the Ethnic Embroidery Image

For data augmentation, traditional methods cannot change their data distribution. The GAN generates image details and local area characteristics in the process of generating images and has great advantages in detail processing. Ethnic embroidery image data has unique ethnic element features and local texture features, which are suitable for data enhancement using GAN. For such images with ethnic element features, the extraction vector of image features should be added to the generative model of GAN as prior knowledge. Then, the generator can simulate the image distribution of the training set and generate real images with mapping relationships through feature constraints [19–21]. In algorithm iterations, the loss function needs to be continuously used to adjust the orientation of the generated image, and the discriminative results can influence the generator to make adjustments to the generated image. The network structure of the GAN is shown in Figure 2.

The first part of the neural network model consists of three Res-Desnet (Resnet) layers, whose purpose is to map features at different times to a space of the same dimension. After the mapping of the Res-Desnet layer, the outputs of different parts are concatenated into a sequence. The second part of the model is a two-layer bidirectional long short-term memory (Bi-LSTM), which is used to analyze the information at the current moment and after the current moment. The third and fourth parts of the model are both Res-Desnet layers.

The mathematical expression of the GAN can be written in the form shown in

(1) $$\begin{array}{c} \underset{G}{\min}\underset{D}{\max}V\left(G,D\right)=E_{x∼p_{\text{data}}\left(x\right)}\left[\log\;D\left(x\right)\right]+E_{z∼p_{z}\left(z\right)}\left[\left.\log\left(1-D\left(G\left(z\right)\right.\right)\right)\right]. \end{array}$$

In equation (1), *D* is the discriminator, *G* is the generator, *x* is the data set, *P*_data_(*x*) is the generated data distribution, and *P*_*Z*_ is the parameter.

CNN can extract features from data. It is a partially connected network. In a fully connected network, all nodes in the input layer are connected to all nodes in the hidden layer. There are many parameters to learn, and the speed is slow. The connected network increases the speed. For the research object, it is more convenient and reliable to use CNN to extract and represent the shallow features of embroidery images. The calculation method of the convolutional layer in the CNN model can be shown in

(2) $$\begin{array}{c} \text{conv}=\sigma \left(iM^{\circ }W+b\right). \end{array}$$

In equation (2), *b* is the weight, *W* is the neural network parameter, *M* is the number of neurons, and *σ* is a nonzero constant.

The features extracted in the shallow CNN can be used as the feature vector of the GAN experiment. In addition, a deconvolution layer needs to be set after each convolution layer. The deconvolution layer can be regarded as the inverse process of CNN. During deconvolution, the image is de-pooled to visualize the image. The deconvolution process is a process without learning and training [22]. Lv and Qiao constructed a cognitive computing system model based on a deep belief network [23]. The visualization process is to verify and display the feature map. The workflow of deconvolution is shown in Figure 3.

In Figure 3, the process of extracting image features by deconvolution is from input to convolution to pooling, and then, the reverse process to visualize the results. Therefore, the CNN is trained in the first stage of the experiment. There is a one-to-one correspondence between the feature map and the local receptive field, and the texture features of the image can be extracted under this one-to-one correspondence. The parameters adjusted during the training process need to consider the effect of feature visualization.

The structure of the GAN is shown in Figure 4.

Traditional GAN generates inefficient, uncontrolled, and unstable training. To improve the network structure in terms of stability, the Conditional Global Area Network (CGAN) appears. The structure of the CGAN is shown in Figure 5.

CGAN has input conditions to both models, which allows the GAN model to generate data by the influence of the conditions. The overall loss function of the CGAN model can be written in the form shown in

(3) $$\begin{array}{c} \underset{G}{\min}\underset{D}{\max}V\left(D,G\right)=E_{x∼p_{\text{das}}\left(x\right)}\left[\log\;D\left(xy\right)\right]+E_{z∼p_{z}\left(z\right)}\left[\log\left(1-D\left(G\left(zy\right)\right)\right)\right]. \end{array}$$

Therefore, according to the existing image information of embroidery data and the feature vectors that have been extracted, the image elements generated by using CGAN with constraints as the experimental model are more in line with the characteristics of embroidery images. The feature vector extracted from the CNN is input into CGAN as a constraint condition, and then, a CGAN data enhancement algorithm under the influence of the ethnic element feature condition appears.

When segmenting the embroidery pattern, first, the embroidery pattern is denoised, binarized, and grayscale processed. Then, the target image is marked with a morphologically connected domain to obtain the initial outline position of the target subimage. Finally, the edge tracking of the CV model is performed on the different subimages on the gray scale pattern to complete the segmentation of the embroidery pattern. The algorithm flow is shown in Figure 6.

The data used in the experiment is the data obtained by own shooting. The length of the image is 831, the width is 677, a total of 5000 images, and the ratio of the amount of experimental data to the amount of training data is 8 : 2. The software configuration used in the experiment is shown in Table 1.

The algorithm firstly de-noises, Otsu binarizes and grayscales the color clothing pattern. Secondly, the target pattern is marked with a morphology connected component (MCC) to obtain the initial contour position of the target subimages. Finally, the Chan-Vase (CV) model edge tracking is performed on different subimages on the gray scale pattern successively to complete the automatic segmentation of ethnic costume patterns.

A two-dimensional *n* × *n*  MCC is an *n* × *n* array composed of *n*^2^ processing units, the structure of which is shown in Figure 6(b). PE(0,0) (processing element) represents the processing unit in the upper left corner of the mesh, and PE(*i*, *j*) represents the processing unit in the *i*th row and the *j* th column of the mesh. Obviously, PE(*i* × *n*, *j*)=PE(*i*, *j*). Each processing unit is a processor that can only perform basic arithmetic and logic operations. All processing units perform corresponding operations in a continuous manner, all control signals are from a single control unit, and each PE is connected to its 4 neighbors. The PEs at the edge are connected to each other, that is, the leftmost PE of each row is connected to the rightmost PE of the row, and the uppermost PE of each column is connected to the lowermost PE of the row. The connection of the interconnection network is unidirectional. In a unit routing, all PEs transmit their data to the PEs directly connected to them in the specified direction.

The Morphology Connected Component Chan-Vase (MCC-CV) algorithm searches for a connected component from the binarized pattern *A*, and the extraction for a single connected component is shown in

(4) $$\begin{array}{c} X_{k}=\left(X_{k-1}⊕\hat{B}\right)\cap A,\;k=1,2,\ldots . \end{array}$$

In equation (4), the meaning of *A* is the target, and *B* is the structure element. *X*_*k*_ is the result of each iteration, *X*_*k*−1_ is the initial position of the connected domain marker. When *X*_*k*_=*X*_*k*−1_, it will not be iterated. The labeling of different blocks is completed one by one through repeated iterations of the morphological processing results.

After the pattern A is marked by the connected domain, a color marking map *C* is formed. The different color marking blocks *Y*_*i*_ in different *C* in the color marking map correspond to a subgraph Ω_*i*_ to be divided in the original pattern, where *i*=1,2,…, *nn* represents the number of subgraphs to be segmented marked by the morphologically connected domain. The marker block *Y*_*i*_ gives the approximate spatial position and size of the subgraph Ω_*i*_ to be divided, so it can be used as the initial outline for the evolution of the CV model. For a subgraph Ω to be divided, the evolution curve *C* can divide the gray scale pattern *I*(*x*, *y*) corresponding to the primitive Ω into foreground Ω_*f*_ and background Ω_*b*_, and *C*_*f*_ and *C*_*b*_ are used to represent the gray value of pixels in the foreground Ω_*f*_ and background Ω_*b*_ areas, respectively. The energy function of the CV model is shown in [24–26]

(5) $$\begin{array}{c} E_{CV}\left(C\right)=E_{CV-\Omega_{f}}\left(C\right)+E_{CV-\Omega_{o}}\left(C\right)=\int_{\Omega_{l}}{\left|I-C_{f}\right|}^{2}\text{d}x\text{d}y+\int_{Q_{b}}{\left|I-C_{b}\right|}^{2}\text{d}x\text{d}y. \end{array}$$

When the evolution curve is at the edge of the pattern element, equation (5) obtains the minimum value, *E*_*CV*_(*C*)=0. Adding the curve length and area energy constraints to equation (5), the expression of the energy functional of the CV model can be shown in

(6) $$\begin{array}{c} E_{CV}\left(C,C_{f},C_{b}\right)=\mu L\left(C\right)+vS\left(C\right)+\lambda_{1}\int_{\Omega_{t}}{\left|I-C_{f}\right|}^{2}\text{d}x\text{d}y+\lambda_{2}\int_{\Omega_{o}}{\left|I-C_{b}\right|}^{2}\text{d}x\text{d}y. \end{array}$$

In equation (6), *L*(*C*) represents the length of the evolution curve *C*, *S*(*C*) represents the area inside the curve *C*, and *μ*, *ν*, *λ*_1_  and *λ*_2_ are the weights of the corresponding energy terms, respectively. In *E*_CV_(*C*, *C*_*f*_, *C*_*b*_), the first two terms are internal constraints, and the curve is kept smooth during the evolution process, and the last term is an external constraint, and the curve is obtained in the evolution process to approximate the edge of the pattern element. The evolution curve *C* is implicitly expressed by the level set *φ*, so the energy functional expression of the level set of the CV model can be rewritten as the form shown in

(7) $$\begin{array}{c} E_{CV}\left(\varphi ,C_{f},C_{b}\right)=\mu \int_{\Omega }H^{\prime }\left(\varphi \right)\left|\nabla_{\varphi }\right|\text{d}x\text{d}y+v\int_{\Omega }H\left(\varphi \right)\text{d}x\text{d}y+\lambda_{1}\int_{\Omega }{\left|I-C_{f}\right|}^{2}H\left(\varphi \right)\text{d}x\text{d}y+\lambda_{2}\int_{0}{\left|I-C_{b}\right|}^{2}\left(1-H\left(\varphi \right)\right)\text{d}x\text{d}y. \end{array}$$

In equation (7), *H*(*φ*) and *H*′(*φ*) are regular approximate representations of Heaviside function and Dirac function, and their expressions are shown in

(8) $$\begin{array}{c} H\left(\varphi \right)=\frac{1}{2}{\left[1+\frac{1}{\pi }\arctan\left(\frac{\varphi }{\varepsilon }\right)\right]}_{0}^{0}, \end{array}$$

(9) $$\begin{array}{c} H^{\prime }\left(\varphi \right)=\frac{1}{\pi }\cdot \frac{\varepsilon }{\varepsilon^{2}+\varphi^{2}}. \end{array}$$

In equation (9), ε is a positive number. Equation (7) is solved according to the variational principle and gradient descent principle, and its partial differential equation is obtained, as shown in

(10) $$\begin{array}{c} \frac{\partial x}{\partial t}=H^{\prime }\left(\varphi \right)\left[\mu \text{div}\left(\frac{\nabla \delta }{\left|\nabla \delta \right|}\right)-v\right]-H^{\prime }\left(\varphi \right)\left[-\lambda_{1}{\left(1-C_{b}\right)}^{2}+\lambda_{2}{\left(1-C_{f}\right)}^{2}\right]. \end{array}$$

The mathematical expression of *C*_*f*_ in equation (10) is shown in

(11) $$\begin{array}{c} C_{f}=\frac{\int_{\Omega }I\left(x,y\right)H\left(\varphi \right)\text{d}x\text{d}y}{\int_{\Omega }H\left(\varphi \right)\text{d}x\text{d}y}. \end{array}$$

The mathematical expression of the GAN is shown in

(12) $$\begin{array}{c} \underset{G}{\min}\underset{D}{\max}V\left(G,D\right)=E_{x∼p_{\text{das}}\left(x\right)}\left[\log\;D\left(x\right)\right]+E_{z∼p_{z}\left(z\right)}\left[\log\left(1-D\left(G\left(z\right)\right)\right)\right]. \end{array}$$

### 3.3. Application of DL in Grassland Cultural Tourism

Tourism commodities are not only a very vital source of economic composition in the tourism industry of the area it sells, but also a good way to promote the culture of this area. The prosperity and development of the tourism commodity industry can drive the economic development of production and life in the grassland area. It can promote a virtuous cycle of economic development in the region, making the economy more developed and the society more stable and harmonious. At the same time, through the sales of different forms of tourism commodities at this stage, the cultural development and history of the local area can be well spread to the hometown of tourists, to make it famous. Although embroidery items are very popular among tourists, they are traditional handicrafts, it is very time-consuming and labor-intensive to make, and the cost is quite high. It cannot be well protected and perfected only by the abilities of some existing old folk artists or individuals. Government support and the introduction and formulation of relevant protection policies all need to keep up with the development of the embroidery industry. The clothing sold in tourist attractions contains the most famous cultural characteristics of the tourist attractions, and most of them are unique local products, which are very local characteristics. If a tourist attraction cannot design and produce unique tourist commodities in its own region, it is difficult for the tourism culture of this region to have a higher and long-term development. With the further development of modern tourism, cultural tourism commodities are more sought after by the people, and the competition in the tourism commodity market has also become the competition of traditional culture. General clothing tourism commodities in tourist attractions are mostly in the form of cultural shirts, shirts, dresses, trousers, handbags, special necklaces, etc., These tourism commodities are easy to carry, easy to produce, cost-effective, and have strong cultural characteristics.

Traditional embroidered clothing and other tourist commodities are not sold much in tourist attractions. Most of them are mainly children's clothing and accessories, and they are mostly handmade by folk artists. The output is small, time consuming, and expensive. However, to attract more tourists and even young tourists to the grasslands to travel and consume, it is more urgent to produce clothing tourism products with modern characteristics. Among the many tourist attractions, printed T-shirts with unique local cultural characteristics and cultural patterns are the most sought. As a representative of modern casual clothing, cultural shirts have outstanding advantages in functionality and portability. It is the most important feature of the tourism products. Most of the costumes for photographing tourist attractions are exaggerated in shape and colorful. The most distinctive local traditional culture is designed and processed in the form of clothing, and it is rented and sold in local commemorative tourist attractions. Tourists can choose their favorite clothing styles and shapes to take pictures and keep them as souvenirs. The photos taken can be kept forever, so that tourists not only keep their beautiful memories during the travel. When they return to their hometowns and share photos with relatives and friends, the local clothing culture will be spread virtually, so that more people can intuitively understand local clothing and cultural characteristics by photography works. This form of clothing is also a kind of clothing tourism commodity. In recent years, this form of clothing has gradually opened and is sold to the tourists, in addition to simply being used as photo style clothing. Through the purchase of clothing tourism products that are different from traditional forms, the local history and culture can be more deeply understood and felt.

Through the basic theory of DL from multi-perspective, the modern inheritance methods, expression methods, and specific design patterns of the digital design of national culture are explored, and the design methods and laws that can be followed and used are summarized, and a database suitable for embroidery craftsmanship is established. The embroidery techniques and stitching methods that are about to be lost are stored for future generations to learn and imitate.

## 4. Design of the Data Enhancement System for Embroidery Images

The application of embroidery images is mainly studied. To apply data enhancement services and style transfer to specific scenarios, a system for data enhancement of embroidery images is designed. The design of prototype system mainly includes three aspects: image acquisition equipment, image processing and storage, and image service and application. It has three main modules. The image acquisition terminal uses professional shooting equipment [27–29], such as cameras and mobile phone terminals with acquisition functions. The function of the acquisition terminal is to transmit the collected embroidery images to the server, and inform the image processing server port of the required service request, and wait for the server to operate, similar to the user using the port. The design of data enhancement system for the embroidery image is shown in Figure 7.

The image processing and storage server in Figure 7 mainly has two functions. On the one hand, it performs data storage and cloud backup to ensure security when receiving a request from the image acquisition terminal. On the other hand, the request is parsed, and the model invocation of the image service application is performed according to the parsed content. The image processing and storage server is composed of multiple server clusters and is directly connected to the cloud storage server, so that the results of processing and feedback can be displayed in a detailed list of operation information for the administrator to view, which also facilitates the later management and optimization of the system. The image service application is mainly the invocation of the application model, and data enhancement will be performed according to the request sent by the image processing terminal. The data generated by the data enhancement service will be stored in the storage server at any time. After the application operation of image data enhancement is completed, the system will perform image evaluation index detection on the generated effect image. Qualified images will be fed back to the storage server, which in turn will inform the image acquisition terminal of the end of the service. The user can know the processing result according to the display of the acquisition terminal. The three modules of the prototype system that are connected to each other not only can send requests, but also can provide feedback of results to each other, and relying on the cloud storage server enables the records to be archived. These measures contribute to management and model improvement.  Figure 8 shows the architecture of the data augmentation system for embroidery images.

The data enhancement system of ethnic embroidery image is divided into four layers. As shown in Figure 8, its functions are as follows: the hardware layer mainly provides hardware support for the system and basic service layer, and provides a powerful graphic processing unit (GPU) support in the process of application services, and store the effect image generated by the service to the cloud server. The storage service of the cloud server runs in the Hadoop environment, which can quickly receive and store images generated by application services and record information for system operations. The basic service layer is mainly to call the service invocation of the application model and use the hardware support of the next layer to perform the service requested by the user. The service model mainly includes data enhancement service model and style transfer application model. The services of the two models are supported by the keras framework, which is divided into a training part and a direct testing phase. The service scheduling layer mainly plays the role of connecting the mobile application layer and the basic service layer. When receiving the request of the mobile application layer, it performs service analysis and transmits it to the basic service layer, and then, schedules the two major application service functions of the system. After the operation is completed, the service scheduling layer can feedback the generated results to the mobile application layer to convey information. The mobile application layer mainly performs image acquisition and preliminary processing based on acquisition device terminal for image collection and preliminary processing. This layer is used to send a request to the service scheduling layer of the system to obtain the service after getting the user's usage request, and display the result after the server's operation ends.

To sum up, the research can be divided into two points. (1) From the perspective of system requirements, a set of application service prototype system for data enhancement and image style transfer of ethnic tie-dye images was designed by means of internet services. The system structure is divided into four layers for design, and the relationship between each layer is used to store, transmit, apply, and display image data. (2) From the perspective of service independence, each module of the application service prototype system for image data enhancement and image style transfer is independently deployed, and the user request is connected with the system service by means of the acquisition terminal and the service scheduling layer. And using the cloud server features, the system model is deployed on the cloud platform as a whole, and the system management performance can be improved through information feedback and recording, thereby saving later maintenance costs. The design and deployment of this prototype system provides a platform example for the inheritance and digital protection of ethnic tie-dye elements. This independent deployment method and the characteristics of cloud storage not only improve the management performance and service performance of the entire system, but also provide full tracking records between users and administrators. The acquisition of record information also facilitates the maintenance of the later platform and system and the expansion of the model. The relationship between the entire system structure and deployment strategy can be used for subsequent research and use.

## 5. Experimental Results and Analysis

### 5.1. Image Extraction and Experimental Results of Visualization

An example of the output image after data enhancement of the ethnic embroidery image is shown in Figure 9.

Figure 9 denotes that the optimized CGAN generates blurred images after 5000 iterations, and the basic color tone has great defects. During the 7000 iterations of the algorithm, the image gradually appeared outline. After 8000 iterations, its personalized features are enhanced, and it is similar to the real dataset to a certain extent. The generated image distribution not only completes the matching of the color tone similarity with the real image, but also presents features such as patterns and textures. The model tends to be in a stable state after 5000 iterations, and the transfer effect of tie-dyed image texture features is better, and symmetrical patterns can be seen. The determination of the boundary makes the goal of migrating the image more specific. Compared with regular images, the transfer effect is better.

The results of the loss function change of the generative model in the optimized CGAN are shown in Figure 10.

Figure 10 refers that the model training is not stable, it has been in a turbulent state before 20000 iterations, and the controllability is extremely poor. After 20000 iterations, it starts to decrease slowly, gradually stabilizes, and stabilizes overall after 25000 iterations. Although the training of GAN is unstable, under the constraint of conditional feature vector, its completion rate and experimental effect are better. Compared with the original model, the concretization of conditions and the extraction of feature constraint rules are meaningful for experiments with less data and a simple structure.

Figure 11 indicates the corresponding relationship between the number of iterations and the peak signal-to-noise ratio (PSNR) value.

PSNR can be used to objectively evaluate the image quality, and the PSNR value must be greater than 30db to prove that the image is above the benchmark. (a) Indicates that the experiment is an object with a relatively clear boundary and (b) shows that the experiment is an object with a relatively unclear boundary. In Figure 11, the PSNR value of the model is 28.21 when the algorithm is iterated 1000 times, the PSNR value of the model is 30.16 when the algorithm is iterated 5000 times, but the PSNR value of the algorithm is 30.22 when the algorithm is iterated 8000 times. The larger the number of iterations of the algorithm, the better the generated image effect. In addition, when the number of iterations of the model exceeds 80000, the image generated by the model reaches the benchmark.

### 5.2. Analysis of Experimental Results of the Automatic Segmentation Algorithm

To analyze the performance of the proposed algorithm, a number of ethnic costume patterns of different complexity are selected and 6 algorithms are used for segmentation, respectively, and the boundary recall (BR) of each segmentation subimage and ground truth is calculated. The number of segmentation subgraphs Num_a_ of each algorithm under different BRs is counted, and *P* is calculated. The experimental results are shown in Figure 12.

Figure 12 expresses that the proposed algorithm MCC-CV realizes automatic segmentation based on the snakes algorithm, and the segmentation effect is significantly better than the other automatic segmentation algorithms. The experimental results show that under the BR of 0.5, the segmentation accuracy of the proposed algorithm is 60%, while the average segmentation accuracy of the other three types of automatic segmentation algorithms is below 20%. Compared with the 19.7% segmentation accuracy of the Clabel automatic segmentation algorithm, the segmentation accuracy of the proposed algorithm is improved by 40%. Under the BR of 0.7, the segmentation accuracy of the proposed algorithm is above 50%.

## 6. Conclusion

Mongolian embroidery is a national intangible cultural heritage and an important treasure in China. In the diversified environment of the world, inheritance and development have always been a significant historical task. To this end, a CGAN based on embroidery image features as constraint rules is proposed and constructed. The texture features of the image are extracted by convolutional layers, and the extracted results are input into the model as conditional vectors. The model can generate images conforming to the embroidery features at a very fast speed by using the embroidery features as prior constraints. And image quality detection and human eye feature judgment are used to perform effect detection on the data-enhanced image of the generated model. An image segmentation algorithm based on MCC-CV is proposed. The algorithm firstly de-noises, binarizes, and grayscales the embroidery image. Secondly, the target pattern is marked with an MCC to obtain the initial contour position of the target subimages. Finally, the CV model edge tracking is performed on different subimages on the gray scale pattern successively to complete the automatic segmentation of embroidery image. The results denote that the proposed algorithm MCC-CV realizes automatic segmentation on the basis of snakes algorithm, and the segmentation effect is obviously better than other automatic segmentation algorithms. The experimental results indicate that when the proposed algorithm meets the BR of 0.5, the segmentation accuracy of the proposed algorithm is 60%, while the average segmentation accuracy of the other three types of automatic segmentation algorithms is below 20%. Compared with the 19.7% segmentation accuracy of the Clabel automatic segmentation algorithm, the segmentation accuracy of the proposed algorithm is improved by 40%. Under the BR of 0.7, the segmentation accuracy of the proposed algorithm is above 50%. However, the proposed algorithm still has many deficiencies, and the proposed GAN parameters have poor controllability. After each adjustment of the parameters, it needs to be trained again, which is a waste of time. Therefore, the method that can guarantee the image quality and stable performance is the future research direction.

## Figures and Tables

**Figure 1:** Representative Mongolian embroidery patterns.

**Figure 2:** The network structure of the GAN. (a) Generative model; (b) discriminative model.

**Figure 3:** The workflow of deconvolution.

**Figure 4:** GAN.

**Figure 5:** The structure of the CGAN.

**Figure 6:** The algorithm flow of MCC-CV algorithm. (a) Algorithm flow; (b) model; (c) pseudocode.

**Figure 7:** The data enhancement system of the embroidery image.

**Figure 8:** The architecture of the data augmentation system for embroidery images.

**Figure 9:** The result of data enhancement of ethnic embroidery image. (a) 2000 iterations; (b) 5000 iterations; (c) 7000 iterations; (d) 8000 iterations.

**Figure 10:** The loss function of the generative model. (a) First test; (b) second test.

**Figure 11:** The corresponding relationship between the number of iterations and the PSNR value. (a) First test; (b) second test.

**Figure 12:** Experimental results of automatic segmentation algorithm. (a) The first test; (b) the second test.

**Table 1:** Experimental indicators of the model.

Items	Indicators
Number	5000
Size of batch	1024
Number of network layers	6
Dropout	0.2
Learning rate	0.1
Optimizer	Adam

## Data Availability

The data used to support the findings of this study are included within the article.
